The article "A Study to Assess the Quality of Reporting of Animal Research Studies Published in PubMed Indexed Journals: A Retrospective, Cross-Sectional Content Analysis" was published in 2022. Journal: Cureus.

# A Study to Assess the Quality of Reporting of Animal Research Studies Published in PubMed Indexed Journals: A Retrospective, Cross-Sectional Content Analysis

**DOI:** 10.7759/cureus.21439

**Published:** 2022-01-19

**Authors:** Kruttika R Chitnis, Ayesha C Shah, Sharmila V Jalgaonkar

**Affiliations:** 1 Pharmacology and Therapeutics, Seth Gordhandas Sunderdas Medical College and King Edward Memorial Hospital, Mumbai, IND

**Keywords:** reproducibility, optimal reporting, experimental, checklist, animal details

## Abstract

Objectives: A complete and concise pre-clinical experimental research gives detailed information about the disease-specific model, prevents duplication, and saves animal life, money, as well as time. It will also allow readers to effectively interpret and evaluate the work and ensure that others can replicate the experiments described. The present study was conducted to assess the adequacy of animal details provided in published experimental animal studies.

Methods: All in vivo studies published as full-text articles in two PubMed indexed journals (one Indian and one international) from January 2011 to December 2019 and satisfying the inclusion norms were included. A checklist consisting of 27 discrete items subdivided under three domains, viz. animal details, disease model, and guidelines, was used. Every article was assessed by two investigators independently for determining the reporting quality.

Results: One hundred and seventy-seven studies satisfied the inclusion criteria. Age or age range was reported in 20.34% of the articles in the Indian journal and 5.88% articles in the international journal (p=0.019). Housing and husbandry details were reported in all the articles published in the international journal and 82.7% of the articles in the Indian journal (p=0.001). The disease/pathology studied was given in 70.62% of articles published in the Indian journal and 86.27% of articles published in the international journal (p=0.029). None of the studies provided details of genetic modification, health status, sample size calculation, steps taken to minimize bias, and implementation of randomization.

Conclusion: There is a need for optimal reporting of certain relevant animal details, disease models, experimental procedures, sample size calculation, and adherence to guidelines by the researchers for which the reporting was found to be sub-par to improve reproducibility and validity of animal research.

## Introduction

Research in science and biomedicine relies highly on preliminary animal experimental studies and investigations. Appropriate descriptions in such studies enable researchers to interpret the data effectively, evaluate and replicate findings, addressing the gaps in knowledge, consequently leading to the advancement of science [1]. Data extrapolated from this research aims to provide a rationale for the hypotheses studied by clinical researchers and epidemiologists. The contribution of animal research to the field of drug discovery and development has resulted in numerous improvements in the medical field [2].

The article "A Study to Assess the Quality of Reporting of Animal Research Studies Published in PubMed Indexed Journals: A Retrospective, Cross-Sectional Content Analysis" was published in 2022. Journal: Cureus.

The difficulties inherent in extrapolating the results of experimental research from animals to man have long been recognized by scientists and pharmacologists [3]. Many animal studies are poorly planned, performed, and analyzed, which is one explanation why animal research has poor translational value in human trials. Moreover, the poor design of studies may expose humans to unnecessary harm [3,4]. Another factor that could be contributing to the inability of animal testing findings to be replicated in humans is that analyses and summaries of animal research evidence are methodologically insufficient, leading to misinterpretation of results and often non-reproducibility. When these studies are published, many critical elements regarding details about animals, conditions under which experiments are performed, and the procedures undertaken are often missing [5]. Consequently, the lack of reproducibility of preclinical studies has been identified as a hindrance to the translation of basic research into effective clinical therapies [6].

The rise of open-access journals has transformed the publishing process, increasing the accessibility of research data from a variety of fields. Nonetheless, details of the experimental research in the published article are often inadequate, leading to the inference that, even if the science is sound, the papers themselves are not always "fit for purpose." Thus many publications prove to be of limited utility as instruments to educate policy, clinical, and scientific practice due to the lack of precise details with crucial information [7]. For the same reason, the Animal Research: Reporting of In VivoExperiments (ARRIVE) guidelines were introduced in the year 2010 to enhance the standard of animal research reporting (although there is a report contrary to that) [8]. ARRIVE guidelines require the authors to stick to a standard format, and despite its widespread endorsement by the scientific community, its impact on the transparency of reporting in animal research publications has been limited [9]. The present study was conducted to assess the adequacy of key details provided in published animal studies in two journals focusing on experimental research.

This article was previously presented as an e-paper presentation at the virtual Pharmacology conference, Andhra Pradesh Association of Pharmacologists Conference (APPSCON) 2020, on 4th December 2020.

The article "A Study to Assess the Quality of Reporting of Animal Research Studies Published in PubMed Indexed Journals: A Retrospective, Cross-Sectional Content Analysis" was published in 2022. Journal: Cureus.

## Materials and methods

Study design

This study was a cross-sectional, retrospective content analysis conducted to qualitatively assess the reporting standard of animal studies. As data was available in the public domain and did not involve retrieving any sensitive data, the study was exempted from the Institutional Ethics Committee review (EC/OA/69/2020).

Data extraction

All experimental animal studies, published in English in all the issues of the two PubMed indexed journals between 2011 and 2019, were downloaded from the respective journal sites. The selection of journals was based on considerations of access and wide coverage of preclinical, experimental research. The two journals did not have a requirement to comply with ARRIVE checklist for submission involving animal research. Selection of eligible articles was made by all three investigators independently by the screening of titles, abstracts, keywords, and methodology to identify original animal research. We excluded review articles, letters to the editor, short communications, in vitro experimental studies, and meta-analyses published in these journals. The final spreadsheet included studies collating the lists of studies by individual investigators.

Assessment of adequacy and quality of reporting

For each original published article reviewed, data collection was done, which contributed information about the reporting quality of the paper. For the purpose of analysis, the investigators brought 27 discrete items nested across three domains, viz. animal details, disease model, and guidelines. The final checklist was validated for its content by 10 experts with experience in the field of animal research. Each item in this checklist had a content validity ratio (CVR) >0.62. For a panel consisting of 10 experts, the minimum CVR should be 0.62 [10]. This checklist was used to assess whether details relating to each of the 27 items (17 for animal details, eight for disease model, and two for guidelines) were mentioned in the published manuscript after giving a thorough read to each article by two investigators independently. Studies explicitly reporting the item or the details about the item of interest in the manuscript, an entry of ‘YES’ was made against the item in the spreadsheet. Details were retrieved through careful reading of the full papers. On the contrary, if the reported information was found to be indistinct or missing altogether in the article, an entry of ‘NO’ was made against that item in the spreadsheet. For example, for reporting of the item ‘sex of the animals,’ three options were taken into consideration viz. ‘male,’ ‘female,’ or ‘either/both’ for which the corresponding entry in the spreadsheet would be ‘YES.’ Similarly, for the item ‘housing and husbandry,’ details regarding environmental conditions (temperature, humidity, light-dark cycle, access to food and water, and the cages used for housing the animals) were considered to make ‘YES’ as the entry against that item in the spreadsheet. Regarding the items pertaining to guidelines, for example, statement of adherence to Committee for the Purpose of Control and Supervision of Experiments on Animals (CPCSEA)/other country-specific guidelines, an explicit statement of adherence, if included in the manuscript, was considered to report a ‘YES.’ Any discrepancies were resolved by reanalysis of studies, and a final decision was reached by discussion and deliberation among all investigators.

The article "A Study to Assess the Quality of Reporting of Animal Research Studies Published in PubMed Indexed Journals: A Retrospective, Cross-Sectional Content Analysis" was published in 2022. Journal: Cureus.

Data analysis

Data were expressed using descriptive statistics like frequencies and percentages. Statistics were applied using IBM SPSS Statistics software, version 25.0 (IBM Corp., Armonk, NY). Categorical data for comparison between the two journals were analyzed using Chi-square or Fisher’s exact tests, and p<0.05 was considered significant.

## Results

Overall, 646 articles from the Indian journal and 97 articles published in the international journal during 2011-2019 were initially screened for suitability. Figure 1 explains the retrieval and selection of articles from the Indian journal for the present study. For the Indian journal, out of the 646 published articles, screening of title and abstracts excluded 469 articles. These 469 articles included review articles, letters to editors, short communications, in vitro experimental studies, and metanalyses. Only 177 animal studies published in the Indian journal were included for the final analysis. For the international journal, out of the 97 articles, 46 articles were clinical studies. Fifty-one animal studies were found eligible and were included to conduct the content analysis (Figure 2). The sequence is summarized in Figures 1, 2.

**Figure 1:** Flow diagram of retrieval and selection of articles from the Indian journal.

**Figure 2:** Flow diagram of retrieval and selection of articles from the international journal.

Animal details

All articles published in either journal mentioned the common name of animals or the species of animals used in the experimental study. The most commonly used experimental animal was rats (81.58%, i.e., 186 out of 228 studies) followed by mice (19.3%, i.e., 44 out of 228 studies). The strain of animals was mentioned in 95.48% of the Indian journal articles and 90.19% of the international journal articles (p=0.90), and none of the articles in either journal mentioned the sub-strain. Of the papers reporting the strain of animals (n=214), 63.16% used Wistar rats, 14.91% used Sprague Dawley rats, and 14.47% used Swiss albino mice as experimental animals. The sex of the animals was reported in 91.53% of the studies in the Indian journal and 84.31% of the studies in the international journal (p=0.041). The age or age range of animals was mentioned in 20.34% of the articles in the Indian journal and 5.88% of the articles in the international journal (p=0.019). The weight of the animals was mentioned in 90.4% and 92.15% of the articles in the Indian and international journals, respectively (p=1.000). The source from which the animals were procured was stated in 51.41% and 58.82% of the Indian and international journal articles, respectively (p=0.43). All articles published in the international journal and 82.7% of the Indian journal articles mentioned the details of housing and husbandry conditions (p=0.001). None of the articles in either journal stated the genetic modification status, genotype, health and immune status of the animals, and the sample size calculation. Whether the animals were drug-exposed or drug-naïve was noted in a single study published in the Indian journal and none of the articles in the international journal. The number of animals utilized in the experimental research was stated by 84.75% of the Indian journal articles and 92.15% of the international journal articles (p=0.246). In comparison, the number of groups in which the animals were divided was mentioned by 87.0% of the Indian journal articles and 94.1% of the international journal articles (p=0.213). None of the articles published in either journal mentioned a statement regarding the implementation of randomization according to the recommendation in the ARRIVE guideline. Table 1 lists the items under this domain.

The article "A Study to Assess the Quality of Reporting of Animal Research Studies Published in PubMed Indexed Journals: A Retrospective, Cross-Sectional Content Analysis" was published in 2022. Journal: Cureus.

**Table 1:** Checklist of items for animal details (Domain A). *Chi-square test, **Fisher's exact test; df: degrees of freedom, ARRIVE: Animal Research: Reporting of In Vivo Experiments

Item No.	Checklist Items	Indian journal		International journal		Pearson Chi-square value	df	p-value
A.	Animal Details	Yes n (%)	No n (%)	Yes n (%)	No n (%)			
1.	Common name of animals/Animal species	177 (100%)	0 (0%)	51 (100%)	0 (0%)	-		-*
2.	Strain of the animals	169 (95.48%)	8 (4.5%)	46 (90.19%)	5 (9.81%)			0.090**
3.	Sub strain of the animals	0 (0%)	177 (100%)	0 (0%)	51 (100%)	-		-*
4.	Sex of the animals	162 (91.53%)	15 (8.47%)	43 (84.31%)	8 (15.67%)	2.27	1	0.132*
5.	Age or age range	36 (20.34%)	141 (79.66%)	3 (5.88%)	48 (94.12%)	5.836	1	0.016*
6.	Weight (mean)	160 (90.4%)	17 (9.6%)	47 (92.15%)	4 (7.85%)			1.000**
7.	Genetic modification status	0 (0%)	177 (100%)	0 (0%)	51 (100%)	-		-*
8.	Genotype	0 (0%)	177 (100%)	0 (0%)	51 (100%)	-		-*
9.	Housing and husbandry	148 (83.62%)	29 (16.38%)	51 (100%)	0 (0%)	9.574	1	0.002*
10.	Source of the animals	91 (51.41%)	86 (48.59%)	30 (58.82%)	21 (41.18%)	0.873	1	0.350
11.	Health and immune status of animals	0 (0%)	180 (100%)	0 (0%)	51 (100%)	-		-
12.	Drug used or drug naïve	1 (0.55%)	176 (99.44%)	0 (0%)	51 (100%)			1.000**
13.	Previous procedure	0 (0%)	177 (100%)	0 (0%)	51 (100%)	-		-
14.	Sample size calculation	0 (0%)	180 (100%)	0 (0%)	51 (100%)	-		-
15.	Sample size (No. of animals utilized for the study)	150 (84.75%)	27 (15.25%)	47 (92.15%)	4 (7.85%)	1.851	1	0.174*
16.	No. of control/ experimental groups	154 (87.00%)	23 (13.00%)	48 (94.11%)	3 (5.89%)	1.982	1	0.159*
17.	Randomization as per recommendation in ARRIVE guidelines	0 (0%)	177 (100%)	0 (0%)	51 (100%)	-		-

Disease model

The disease or the pathology under research was given in 70.62% of the Indian journal articles and 86.27% of the international journal articles (p=0.029). All articles published in either journal stated the rationale for conducting the animal study, whereas the rationale for selecting a particular species of animals to address the specific scientific objective was reported by none. The experimental model used to study the disease of interest was mentioned in 45.76% of the articles published in the Indian journal and 56.86% of the articles in the international journal (p=0.203). Whether the intervention was therapeutic or prophylactic was stated in 95.48% of the articles published in the Indian journal and all the articles published in the international journal (p=0.204). The rationale for the procedure was noted in all the articles in both journals. None of the articles commented on the measures taken to minimize bias. Table 2 lists the items under this domain.

**Table 2:** Checklist of items for disease model (Domain B). *Chi-square test, **Fisher's exact test; df: degrees of freedom

Item No.	Checklist Items	Indian journal		International journal		Pearson Chi-square value	df	p-value
B.	Disease Model	Yes n (%)	No n (%)	Yes n (%)	No n (%)			
1.	Disease/pathology studied	125 (70.62%)	52 (29.38%)	44 (86.27%)	7 (13.73%)	5.058	1	0.025*
2.	Rationale for using animals	177 (100%)	0 (0%)	51 (100%)	0 (0%)	-		-
3.	Rationale for the species of animals selected to address the scientific objective	0 (0%)	177 (100%)	0 (0%)	51 (100%)	-		-
4.	Outcome measures selected to address the scientific objective	177 (100%)	0 (0%)	51 (100%)	0 (0%)	-		-
5.	Experimental model	81 (45.76%)	96 (54.24%)	29 (56.86%)	22 (43.14%)	1.954	1	0.162*
6.	Intervention tested-Therapeutic or prophylactic	169 (95.48%)	8 (4.52%)	51 (100%)	0 (0%)			0.204**
7.	Procedure	177 (100%)	0 (0%)	51 (100%)	0 (0%)	-		-
8.	Statement regarding measures taken to minimize bias	0 (0%)	177 (100%)	0 (0%)	51 (100%)	-		-

Guidelines

About 51.97% of the studies published in the Indian journal and 72.55% of the studies published in the international journal mentioned a statement regarding adherence to CPCSEA or any other country-specific relevant guidelines during the execution of the experiments (p=0.010). In comparison, the statement of adherence to the Organisation for Economic Co-operation and Development (OECD) guidelines was mentioned by 25.55% of the studies in the Indian journal and 43.14% of the studies in the international journal (p=0.022). Table 3 lists the items under this domain.

The article "A Study to Assess the Quality of Reporting of Animal Research Studies Published in PubMed Indexed Journals: A Retrospective, Cross-Sectional Content Analysis" was published in 2022. Journal: Cureus.

**Table 3:** Checklist of items for guidelines (Domain C). *Chi-square test, **Fisher's exact test; df: degrees of freedom, CPCSEA: Committee for the Purpose of Control and Supervision of Experiments on Animals, OECD: Organisation for Economic Co-operation and Development

Item No.	Checklist Items	Indian journal		International journal		Pearson Chi-square value	df	p-value
C.	Guidelines	Yes n (%)	No n (%)	Yes n (%)	No n (%)			
1.	Statement of adherence to CPCSEA/other country-specific guidelines	92 (51.97%)	85 (48.02%)	37 (72.55%)	14 (27.45%)	6.820	1	0.009*
2.	Statement of adherence to OECD guidelines	45 (25.42%)	132 (74.58%)	22 (43.14%)	29 (56.86%)	5.987	1	0.014*

## Discussion

This study was conducted to assess the standard of reporting requisite experimental animal research details in published articles. For this study, we chose to narrow our focus to three important domains operationalized as 27 discrete items as they are relatively easily implemented, recommended by current guidelines, and can be unambiguously reported in a manuscript. This study complements existing checklists and stresses the specific information that should be included in research publications of animal studies.

Age, sex, weight, source, genetic nomenclature, microbial/pathogen status, preparation, and assignment (including control groups) are the key information considering any experimental animal study. The availability of specific details for these basic variables in the publication is crucial for enabling replication. Sex influences numerous biological outcomes. Both age and body weight (with ranges) are critical parameters to provide for all animal studies. Age alters many biological outcomes and affects lesions, disease course, physiologic state, and response to experimental variables. Many publications, especially those that involve rat and mouse models, indicate body weight instead of age. Body weight is not identical to age; the correlation is highly dependent on the animal's life stage, stock, and strain. In addition, a variety of husbandry, dietary, and environmental factors have a significant impact on body weight, often through interactions that are poorly understood. Weight, along with age, is vital to include in the animal description because it correlates with numerous biological outcomes. Precise information about genetic modification or genotype becomes imperative in certain areas of research where strains with specific genetic manipulation/mutation (e.g., knock‑out or transgenic) are used [4,5]. For example, the Zucker rat strain, which bears a mutation in the leptin receptor gene, is sugar metabolic deficient and insulin resistant and thus, serves as a spontaneous genetic obesity model. The spontaneously hypertensive rat (SHR) has been the most widely studied model of hypertension, as indicated by the number of publications on it [11].

The article "A Study to Assess the Quality of Reporting of Animal Research Studies Published in PubMed Indexed Journals: A Retrospective, Cross-Sectional Content Analysis" was published in 2022. Journal: Cureus.

The definition of the phrase specific pathogen-free (SPF) is challenging for investigators when characterizing the health/immune/microbial condition of their animals. There is no universal agreement on which agents constitute pathogens and which should be avoided in certain sorts of research or for specific species. The use of the term SPF and determining pathogen exclusion status in genetically engineered laboratory rats are particularly difficult. These animals are vulnerable to immune function dysregulation, which might result in sensitivity to opportunistic infections and hence impact study outcomes [1].

Exploratory content analysis of the in vivo animal research published in the two journals in the present study revealed that only a few articles mentioned the age range (~20% from the Indian journal and ~6% from the international journal). In contrast, the characteristics like sub-strain, genetic modification and genotype, and health and immune status of animals were stated in none of the articles from both journals. Information about the source of procurement of animals was skipped in almost half the articles in the Indian journal and ~40% in the international journal. Assignment of animals to negative or positive control or various experimental groups was described in a high proportion of research articles in both journals (87% and 94% articles in the Indian and international journal, respectively). The majority of the studies also mentioned the species, strain, sex, and weight of animals utilized for the experiment in the published manuscript. In a study by Bara et al. to assess the methodological quality of animal research in critical care, the pre-specified primary outcome was the composite of three animal characteristics: strain, sex, and weight or age [12].

The article "A Study to Assess the Quality of Reporting of Animal Research Studies Published in PubMed Indexed Journals: A Retrospective, Cross-Sectional Content Analysis" was published in 2022. Journal: Cureus.

Details about housing and husbandry of animals were mentioned in all the articles in the international journal, while 16% of the articles published in the Indian journal did not mention these details. Effective reporting of animal research environment includes adequate information about the micro- and macro-environment, diet, water, and housing as these are the potential sources of variation in many studies. A detailed description of food and feeding methods, frequency, and method of providing the feed and water (e.g., ad libitum vs. portioned) is preferable to enable other investigators to effectively assess and reproduce the research. Appropriate descriptions of housing convey the physical, microbial, and social features of the animals' proximate environment. Multiple factors in the animal facility can influence study results, and not all of them can be covered in detail in the materials and methods section. However, at a minimum, the description in the materials and methods section can specify the type of diet, housing, bedding, water, and general environmental parameters (e.g., temperature, humidity, lighting) with appropriate ranges [1].

Optimal reporting of experimental research upholds the reporting of essential details related to the experimental design viz. the disease/pathology studied, the experimental model and outcome measures selected to address the scientific objective, number of animals (sample size), and the sample size calculation, the steps taken to minimize bias, randomization and blinding for improving the validity of animal research [5]. In the present study, most articles published in both the journals mentioned the disease/pathology studied, whereas only about half the studies (45.76% and 56.86% in the Indian and the international journal, respectively) mentioned details about the experimental model. According to a study conducted in China by Zhao et al., 41% of studies did not state the hypothesis or objective of the study as well as the number of animals used in the study [13]. For research studies including animal research, providing sample size information with calculation is very crucial as, if a researcher selects a smaller number of animals, it may lead to missing any significant difference even if it exists in population and if more number of animals selected then it may lead to unnecessary wastage of resources and may lead to ethical issues [14].

Additional relevant details regarding animals and disease model desirable to be stated in the manuscript are the rationale for the procedure, including acclimatization prior to experiments, the rationale for selecting the species for studying the disease/pathological process, whether the intervention being studied is intended for therapeutic or prophylactic use, if the animals were drug naïve or if any previous procedure was done [4,9,15]. In scenarios wherein the animals have been used in more than one study, it is essential to specify the nature of previous use, explaining how the animals were chosen for reuse and assigned to the current study [1].

The article "A Study to Assess the Quality of Reporting of Animal Research Studies Published in PubMed Indexed Journals: A Retrospective, Cross-Sectional Content Analysis" was published in 2022. Journal: Cureus.

Reporting relevant information regarding the disease/pathology and experimental model being used to study the same is necessary for the reproducibility of research. Sufficient information specifying the procedure is a must because there may be numerous approaches for conducting a study; thus, it is important to specify relevant details of the chosen procedure. The description of habituation methods such as acclimatization is crucial in animal research as transportation from one place to another can be stressful for animals, and they need to be kept in a stable environment for a certain period so that they get stabilized in the novel environment prior to conducting any experimental procedure. Failure to become accustomed to the research setting, experimental procedures, and equipment can significantly impact study results [1,4,15].

The risk of bias is a major threat to internal validity. In in vivostudies, selection bias arises when non-random factors impact the distribution of animals to study interventions. Selection bias occurs when identified differences between groups in a study are due to a confounder rather than interventions. Randomization is the best method for evenly distributing confounders across the intervention groups [14]. In this study, none of the articles from either journal mentioned about randomization procedure in the manuscript. In 2010, the Animal Research: Reporting of In Vivo Experiments (ARRIVE) guidelines were developed to improve the transparency and reproducibility of animal studies. ARRIVE guidelines recommend reporting blinding and randomization procedures, i.e., any steps taken to limit the effects of subjective bias when allocating animals to treatment in the study design [5,15,16].

The CPCSEA provides guidelines for performing ethical experiments on animals and maintaining the animal house [17]. Those involved in animal experimentation in India must follow all the existing regulations mentioned in these guidelines while other countries lay down their country-specific guidelines for the execution of animal experiments, e.g., guidelines issued by the Korean National Institute of Health [4,17,18]. In the present study, the housing, care, and experimentation on animals, whether carried out in accordance with the CPCSEA guidelines, was reported by almost half the articles in the Indian journal and above 70% of articles in the international journal. Novel molecules used in the experimental studies may have some toxicological effects, so as per statutory requirements, safety needs to be evaluated in rodents and non-rodents before phase I and phase II clinical trials for acute toxicity [4]. In the present study, only 25% and 43% of articles published in the Indian and international journals, respectively, mentioned testing the safety of the experimental compounds according to OECD guidelines for acute toxicity testing.

The article "A Study to Assess the Quality of Reporting of Animal Research Studies Published in PubMed Indexed Journals: A Retrospective, Cross-Sectional Content Analysis" was published in 2022. Journal: Cureus.

The ability to interpret, evaluate, and reproduce biomedical and other types of laboratory animal research and testing is a reasonable minimum standard for assessing effective reporting in research articles. Authors of in vivo research should make a sincere effort towards the optimal reporting of all relevant scientific details while submitting the manuscript to the journal. Journal editors can substantially contribute to achieving this standard by articulating clear policies and criteria for their authors and reviewers. Improving the quality of publications will also facilitate systematic reviews, thereby generating new knowledge through the synthesis of evidence without using animals. This will also reduce the risk of the researchers being unable to respond to journals' requests for more observations in an experiment, which can lead to manuscript rejection, wasting both animal lives and human resources.

Our study has several limitations: The included articles varied in study outcomes, animals used, and disease types. Some studies may have failed to mention some methodological details when these were employed while executing the study. The purpose of this study was only to assess the reporting quality of studies and did not seek to evaluate the quality of the studies. Lastly, a potential limitation of our study is that it included published articles from only two PubMed indexed journals. More journals would have given the study a broader coverage and boosted its generalizability.

## Conclusions

Overall, this study demonstrated good reporting quality and completeness of details for certain parameters in both the journals like species, strain, sex, weight, housing, number of animals utilized, number of experimental/control groups, disease/pathology studied, outcome measures, nature of intervention and details of procedures. However, some important factors which were poorly reported were age, source of procurement, genetic modification, health and immune status, whether drug naïve, a previously conducted procedure (if any), determination of sample size, experimental model, steps taken to minimize bias, randomization done as recommended in ARRIVE, and acute toxicity studies as per OECD guidelines. A significant difference between the two journals was observed for factors like age, housing and husbandry conditions, disease/pathology studied, and adherence to CPCSEA and OECD; the International journal being better for all the mentioned factors except the age of animals. As journals have a crucial role in improving the standard of research reporting, a statement could be included in the "instruction to authors" section for manuscript submission.
